# The Efficacy of *Harpagophytum procumbens* (Teltonal) in Patients with Knee Osteoarthritis: A Randomized Active-Controlled Clinical Trial

**DOI:** 10.1155/2021/5596892

**Published:** 2021-10-19

**Authors:** Hamid Reza Farpour, Najme Rajabi, Bahareh Ebrahimi

**Affiliations:** ^1^Bone and Joint Diseases Research Center, Department of Physical Medicine and Rehabilitation, Shiraz University of Medical Sciences, Shiraz, Iran; ^2^Shiraz Geriatric Research Center, Shiraz University of Medical Sciences, Shiraz, Iran; ^3^Student Research Committee, Department of Physical Medicine and Rehabilitation, Shiraz University of Medical Sciences, Shiraz, Iran

## Abstract

**Purpose:**

The high prevalence of knee osteoarthritis (KOA) is a major cause of disability among elders. NSAIDs are recommended to reduce KOA patients' symptoms, but their adverse side effects limit their consumption. In this study, we evaluated the effectiveness of *Harpagophytum procumbens* compared to a routine NSAID (meloxicam) on pain reduction and functional improvement of KOA patients. *Patients and Methods*. Sixty patients aged 40–60 years, with painful knee osteoarthritis (grades 1-2 of Kellgren–Lawrence scale) for at least one month, were randomized into two groups with different routine medication periods. Group A consisted of daily administration of two *Harpagophytum procumbens* (Teltonal) tablets (2*∗*480 mg) for one month, and group B consisted of daily administration of meloxicam (15 mg) for ten days. The visual analogue scale (VAS), Western Ontario McMaster University Osteoarthritis Index (WOMAC), Oxford Knee Scale (OKS), and patient satisfaction were evaluated at the baseline and after 2, 4, and 8 weeks.

**Results:**

There were no statistically significant differences between demographic characteristics, pain intensity, and function scores before the treatment. VAS, OKS, and WOMAC scores improved in both groups (*p* < 0.001) over time, but no significant superiority was shown; after 8 weeks: VAS (Teltonal (4.80 ± 1.80) vs. meloxicam (5.06 ± 1.43)), OKS (34.06 ± 4.38, 34.00 ± 7.87, Teltonal vs. meloxicam, respectively), and WOMAC scores (25.73 ± 10.11 Teltonal vs. 26.20 ± 13.94, meloxicam).

**Conclusion:**

Teltonal is an effective and safe treatment in patients with mild KOA in the short term. However, no significant superiority was shown in using Teltonal or meloxicam, in people who cannot take NSAIDs, it can be a good alternative, although difference in medication periods should be considered.

## 1. Introduction

Osteoarthritis (OA) is a progressive joint disease, and knee OA, which accounts for 83% of total OA, is the most common cause of disability among older adults worldwide [1]. In 2017, more than 300 million hip and knee osteoarthritis cases had been reported worldwide, and this prevalence is expected to rise even further in the future, particularly among women [2, 3]. OA management entails pharmacological and nonpharmacological approaches; traditional management of OA focused on the treatment of symptoms associated with the disease, such as pain and physical dysfunction, which focuses on short-term pain control [4–7]. Nonsteroidal anti-inflammatory drugs (NSAIDs) are prescribed to approximately 65% of patients because of their analgesic and anti-inflammatory effects; these drugs are typical options for knee OA treatments, but there is controversy about their role; these medications can be costly or carry substantial side effects, especially in older adults [8–12]. Using NSAIDs in patients with knee OA is associated with gastrointestinal, cardiovascular, and renal complications [13].

Adverse effects of these drugs have caused the patients to look for out-of-standard treatments such as herbal and nutritional supplements, acupuncture, and exercise [7, 14–16]. Meloxicam, as a new nonsteroidal anti-inflammatory drug, has been developed for osteoarthritis and rheumatoid arthritis treatment [17]. This drug contains minor side effects such as abdominal pain and vomiting or severe side effects such as ulceration and bleeding [13, 18, 19]. NSAIDs inhibit cyclooxygenase (COX)‐1 and COX‐2 to varying degrees; also, finding herbal anti-inflammatory drugs which have properties similar to COX inhibitors can be effective in treating inflammations such as osteoarthritis, chronic musculoskeletal pain, and rheumatoid arthritis [10, 18].

*Harpagophytum* or Devil's claw, which was recently introduced under the Teltonal name, is a herbal analgesic with anti-inflammatory effects; this drug is commonly used to treat inflammations such as musculoskeletal pain and rheumatism [20, 21]. The role of *Harpagophytum procumbens* on COX has been shown in different studies [22–24]. For example, in a study by Abdelouahab and Heard, it was shown that using active components of *Harpagophytum procumbens* would reduce COX-2 expression in freshly excised porcine skin [25]. Healthy donors whole-blood assay demonstrated that *Harpagophytum procumbens* inhibits indistinctively COX-1 and COX-2 activity, 37.2 and 29.5%, respectively [24]. Further studies in order to find out the molecular targets of the anti-inflammatory *Harpagophytum procumbens* assert that *Harpagophytum procumbens* prevents the induction of proinflammatory gene expression by blocking the AP-1 pathway [22]. In this regard, one study had evaluated the role of *Harpagophytum* (2,610 mg per day) in comparison with diacerein (100 mg per day four) during four months for treatment of knee and hip OA. This study showed that *Harpagophytum* was as effective as diacerein [21]; in another study, it was revealed that using *Harpagophytum* for eight weeks could improve back pain between 50% and 70%, and also, its effect on hip and knee pain was more than back pain [26].

Many studies have examined the role of *Harpagophytum* in OA treatment [21, 22, 26, 27]; however, there is no new survey to assess the role of *Harpagophytum* in comparison to routine NSAID drugs in knee OA in the short term. This study aimed to compare the efficacy of *Harpagophytum procumbens* (Teltonal) (2*∗*480 mg) with meloxicam (15 mg) in reducing pain and improving the function of patients with knee OA.

## 2. Methods

### 2.1. Study Design

This study was a double-blind, randomized clinical trial approved by the Ethics Committee of Shiraz University of Medical Sciences (ethics number: IR.SUMS.MED.REC.1398.271); also, the protocol was registered at the Iranian Clinical Trial Center with the code of IRCT20191031045291N1. The sample size was determined based on statistical analysis (using the below formula) and taking into account the information of the same study with a conflict interval of 95%, power of 85%, and the probable drop rate of 20%. The sample size in each group was determined 30 (each knee was considered as a sample).

(1) $$\begin{array}{c} n=\frac{{\left(Z1-\left(\alpha /2\right)+Z1-\beta \right)}^{2}sd^{2}}{d^{2}}. \end{array}$$

### 2.2. Participants

Participants included people aged 40–60 years who were referred to physical medicine and rehabilitation clinics of Shiraz University of Medical Sciences (Imam Reza Clinic, Chamran and Rajaie Hospitals); the patients were diagnosed with osteoarthritis by a physiatrist. The details of the intervention were explained to the patients, and only the volunteers participated in the study; the participants were given a consent form to sign, and then, with attention to inclusion and exclusion criteria, the study was conducted. The consort flowchart of this research is shown in Figure 1.

After signing the consent form, patients aged 40–60 years, with pain and other clinical signs of knee osteoarthritis for at least within last month, without any disease around the relevant joint, and with grade 1 or 2 of Kellgren–Lawrence radiographic criteria were included into the study. The Kellgren–Lawrence grading system is a radiological classification of knee osteoarthritis graded from 0 to grade IV; grades 1 and 2 mean doubtful narrowing of joint space and osteophytes [28, 29].

Exclusion criteria were severe grade of knee osteoarthritis based on radiology image (grades III and IV based on Kellgren–Lawrence radiology criteria), patients with knee replacement, history of trauma, and joint fracture injections in or around the affected joint in the last three months and active lumbosacral radiculopathy, collagen vascular diseases such as rheumatic diseases, lupus, and gout, hemorrhagic diseases, consummation of anticoagulants, warfarin, and ticlopidine, nerve damages and neuropathies, infection with *Brucella*, history of allergies and allergic reactions to the drugs, gastrointestinal disorders and stomach problems disorders, other disorders such as diabetes, uncontrolled hypertension, cancer, and significant liver, kidney, heart, and lung disasters, and pregnancy and lactating.

### 2.3. Intervention

The patients were divided into two groups using a block randomization list; treatment of group A consisted of daily administration of two *Harpagophytum procumbens* (Teltonal®, BEHESTAN BEHDASHT Co, Tehran, Iran) tablets (2*∗*480 mg) for one month [30] and that of group B consisted of daily administration of 15 mg of meloxicam (Farabi International Campus®, Isfahan, Iran) as a safe and effective NSAID in the treatment of osteoarthritis (OA) [31] for ten days. In both groups, lifestyle modification and proper knee exercises were taught. Both groups were warned about the possible side effects of the drugs. Contact numbers were given to all patients to consult with researchers, and the symptoms were followed up by the team; patients with gastrointestinal problems had prescribed omeprazole fasting in the morning.

### 2.4. Outcomes

After evaluating for inclusion and exclusion criteria, patients who were enrolled in the study were asked to fill the visual analogue scale (VAS) [32], Western Ontario and McMaster Universities Arthritis Index (WOMAC) [33], and Oxford Knee Scale (OKS) [34] standard questionnaires at the beginning of the study and in the second, fourth, and eighth weeks. To maintain the blinding, the questioner and the data analyzer did not know about the treatments and the patients.

VAS evaluates the pain intensity with 10 degrees (0–10) (Figure 2) [32]. WOMAC is an index to assess the patients' function with three parts: first daily functioning-pain (5 items), second pain, in various daily activities-joint dryness (2 items), and the third part, physical function, by assessing the lameness (17 items). WOMAC total score contains 24 items, and each item includes five scales (0–4). The total WOMAC score is 0–96; ninety-six means the worst function, and WOMAC score reduction means improving [34]. The OKS contains 12 items with five scores from 0 to 4. This questionnaire evaluates the ability to perform various activities function and score 0 and the worst function to 48, the best performance; therefore, increasing OKS score means improvement [33]. Patient satisfaction assessment showed greater quality of care and better treatment outcomes.

### 2.5. Statistical Analysis

The mean change (before and after the intervention) for each criterion was significantly compared with the *t*-test and chi-square using SPSS statistical software. Temporal variations between the two groups were compared by repeated-measures analysis of variance and RM ANOVA.

## 3. Results

### 3.1. Patients' Demographic Data

In this study, 60 knees were evaluated. Given the inclusion and exclusion criteria, 38 knees were included in the study. They were randomly divided into two groups: A (Teltonal group) with 20 knees and group B (meloxicam group) with 18 knees. Eight patients were excluded from the study during the follow-up period; finally, 15 knees from each group were studied. The demographic data are given in Table 1. There was no significant difference between the patients' sex, age, and BMI in each group (Table 1).

Regarding the VAS pain score, there was no significant difference in pain between the two groups before the treatment and in 2, 4, and 8 weeks after the follow-up. Data analysis showed that the rate of pain reduction over time was significantly significant in both groups (*p* value <0.001) (Table 2).

Assessing the patients' performance score in the evaluation was done using the OKS questionnaire. The mean score was 27.6 (13–40) and 27.00 (16–40) in groups A and B. After treating the knee, no statistically significant difference was shown between the groups in the second, fourth, and eighth weeks after treatment. Still, the rate of improvement in performance over time in both groups was significant (*p* value <0.001) (Table 3).

The mean total score of WOMAC in the Teltonal and meloxicam groups, before treatment, was 41.93 (9–64) and 43.13, respectively (13–68). Treatment decreased the mean in both groups in the second, fourth, and eighth weeks of treatment, but the reductions were not statistically significant. The improvement in the overall performance score based on the WOMAC questionnaire was significantly different in both groups over time (*p* value <0.001) (Table 4).

At the end of the eighth week, both groups had a high level of satisfaction with the treatments, and there was no significant difference between the two groups (*p* value: 0.18). During the treatment, only one patient in the Teltonal group complained of fullness in the stomach after taking the drug. Two patients in the meloxicam group complained of stomachache, which was relieved by omeprazole (data not shown).

## 4. Discussion

Osteoarthritis (OA), such as knee OA, as the most common form of arthritis, affects people, especially the elderly, and the OA-induced disability among the patients can influence their life [35]. Patients with OA are likely to be treated with several different pharmaceuticals and nonpharmaceutical interventions. In the long term, finding treatments with fewer side effects and less cost can help them [4, 7, 36]. The results of this study showed that both therapies, Teltonal (2*∗*480 mg/day) and meloxicam (15 mg/day), had acceptable efficacy in treating the disease despite their different consumption period, and a statistically significant difference was observed over time in these two groups in the eighth week after treatment, compared to the beginning of the treatment.

The findings showed that using Teltonal for one month could significantly affect VAS, OKS, and WOMAC scores similar to 10 days' use of meloxicam. Evidence suggests that medicinal herbs can manage OA knee pain due to their anti-inflammatory, antinociceptive, and chondroprotective properties [37–40]. For example, using three yellow oil formulations showed relieving knee pain, and these oils had been considered as alternatives for treatment OA symptomatic due to their inhibitory role on COX and lipoxygenase (LOX), as well as cytokine release [37]. Various studies have been conducted on the role of *Harpagophytum procumbens* on different types of pains, such as the neuropathic, arthritic, hip, knee, or even low back pain in both humans and animals [41–44]. For example, in a study, it was found that patients with chronic low back pain were less likely to use tramadol as a pain reliever in the *Harpagophytum procumbens* extract group than patients in the placebo group. This study showed that at the end of the 3 week experience, 17.6% of the patients who had taken the *Harpagophytum procumbens* extract entirely recovered. In contrast, in the placebo group, 1.8% of patients remained utterly painless [41]. In a systematic review in 2008, twenty-eight clinical trials were identified, and their data analysis showed the efficacy of *Harpagophytum procumbens* [45]. Studies also have shown that the effect of meloxicam, as an inhibitor of COX-2 isozyme, initiates after three days and can impact the WOMAC and VAS, which agrees with our study [29, 46].

As to the role of *Harpagophytum procumbens* on pain scores, few studies have assessed these factors [27, 47, 48]. Wegner et al. used Devil's claw extract for 12 weeks to treat 75 patients with osteoarthritis of the pelvis and knee; the results of their study showed a significant reduction in pain and other symptoms of osteoarthritis [27]. The overall reduction rate of the WOMAC questionnaire was 22.9%, that of the pain score of the WOMAC questionnaire was 23.8%, that of the dryness score was 22.2%, and the fall in the activity restriction score was 23.1%. In this study, the VAS score was also evaluated, and the overall pain reduction of the patient was reported to be 24.5% [27]. These results are in line with the findings of our study. In another study, investigating the effects of *Harpagophytum procumbens* (Devil's claw) on the sensory, motor, and vascular mechanisms of muscle pain showed highly significant improvement of the visual analogue scale after four weeks of treatment with 2 × 480 mg/day of *Harpagophytum* extract [47]. A study by Yocum and his colleagues assessing the role of meloxicam in OA patients showed that meloxicam could significantly affect 4 WOMAC parts [31].

Comparing the efficacy of these two drugs with each other did not show any statistically significant difference between these two groups over time; the differences were not demonstrated in pain scales. Chantre et al. in 2000 compared the efficacy and tolerability of *Harpagophytum procumbens* on 122 patients with knee and pelvic osteoarthritis compared with diacerein. This study showed that this plant was an effective therapeutic agent in treating osteoarthritis, and there was no difference in the efficacy of these two treatments [21]. In another study, a comparison between Doloteffin, a proprietary extract of *Harpagophytum*, and rofecoxib, a selective inhibitor of cyclooxygenase-2 (COX-2), did not show any significant intergroup differences in low back pain patients [49]. There are other studies that indicate using *Harpagophytum procumbens* could affect pain and reduce the patients' need for NSAIDs [48].

The mechanism of action of *Harpagophytum procumbens* has not been fully elucidated, but its role has been demonstrated in blocking the AP-1 pathway, inhibiting COX in blood cells or enhancing CB2 receptor expression and downregulating PI-PLC *β*2 in synovial membranes [22, 24, 25, 50].

Some gastrointestinal side effects such as nausea and vomiting, which occur sporadically, have been reported [13, 18, 19]; our results showed that no severe drug side effects were observed. The limitations of our study included the short-term follow-up, although using NSAIDs for long term is not very common, but we can follow the patients for longer benefits or side effects, assessing the drug plasma level, evaluating the effects of interventions, and using a placebo group. As we know, using a larger sample size assessing the inflammatory biomarkers can confirm our results.

## 5. Conclusion

We can conclude that *Harpagophytum procumbens* (Teltonal drug) is an effective and appropriate treatment for pain reduction and function improvement in patients with mild KOA in short-term. This drug can be a good substitute for NSAIDs although any significant superiority between these two was not shown and the side effects in both groups were not serious.

## Figures and Tables

**Figure 1:** Consort flowchart of the trial.

**Figure 2:** Visual analogue scale (VAS) score pain degrees.

**Table 1:** Demographic data in Teltonal and meloxicam groups.

		Meloxicam group	Teltonal group
Sex	Woman (%)	81.8 (12)	72.7 (12)
	Man (%)	18.1 (3)	27.3 (3)

Age (year (mean ± SD))		55.93 ± 8.54	47.13 ± 5.90
BMI (kg/m^2^ (mean ± SD))		24.26 ± 1.02	26.47 ± 1.71

BMI, body mass index; SD, standard deviation.

**Table 2:** Comparison of the VAS scale in Teltonal and meloxicam groups.

VSA scale	Time	Teltonal (mean ± SD)	Meloxicam (mean ± SD)	*P* value (between groups)
	Baseline	7.13 ± 2.23	7.8 ± 1.30	0.48
	2^nd^ week	5.20 ± 2.14	6.00 ± 1.69	0.26
	4^th^ week	4.7 ± 02.10	5.73 ± 1.57	0.15
	8^th^ week	4.80 ± 1.80	5.06 ± 1.43	0.26

*P* value (within groups)		0.001	0.001	

VAS, visual analogue scale; SD, standard deviation.

**Table 3:** Comparison of the OKS scale in Teltonal and meloxicam groups.

OKS scale	Time	Teltonal (mean ± SD)	Meloxicam (mean ± SD)	*P* value (between groups)
	Baseline	27.6 ± 7.68	27.00 ± 7.25	0.82
	2^nd^ week	32.20 ± 6.24	33.86 ± 6.12	0.46
	4^th^ week	34.4 ± 4.46	33.9 ± 7.73	0.84
	8^th^ week	34.06 ± 4.38	34.00 ± 7.87	0.97

*P* value (within groups)		0.001	0.001	

OKS, Oxford Knee Scale; SD, standard deviation.

**Table 4:** Comparison of the WOMAC scale in Teltonal and meloxicam groups.

WOMAC scale	Time	Teltonal (mean ± SD)	Meloxicam (mean ± SD)	*P* value (between groups)
Total score	Baseline	41.93 ± 13.79	43.13 ± 15.97	0.67
	2^nd^ week	30.66 ± 9.64	27.33 ± 10.36	0.50
	4^th^ week	24.93 ± 8.76	27.46 ± 15.31	0.57
	8^th^ week	25.73 ± 10.11	26.20 ± 13.94	0.23
*P* value (within groups)		0.001	0.001	
Pain	Baseline	10.00 ± 3.07	10.46 ± 2.99	0.67
	2^nd^ week	6.8 ± 2.51	6.26 ± 1.79	0.50
	4^th^ week	5.00 ± 2.09	6.20 ± 3.52	0.57
	8^th^ week	5.06 ± 2.34	6.20 ± 2.75	0.23
*P* value (within groups)		0.001	0.001	
Stiffness	Baseline	1.80 ± 1.74	1.53 ± 1.55	0.68
	2^nd^ week	1.24 ± 1.13	1.48 ± 1.06	0.65
	4^th^ week	0.93 ± 0.96	1.09 ± 0.73	0.40
	8^th^ week	1.00 ± 1.00	1.09 ± 0.73	0.41
*P* value (within groups)		0.09	0.02	
Function	Baseline	30.13 ± 10.40	31.13 ± 12.26	0.81
	2^nd^ week	22.73 ± 7.26	20.00 ± 8.34	0.34
	4^th^ week	18.40 ± 6.64	20.53 ± 11.83	0.54
	8^th^ week	19.66 ± 7.45	19.26 ± 11.41	0.91
*P* value (within groups)		0.01	0.001	

WOMAC, Western Ontario and McMaster Universities Arthritis Index; SD, standard deviation.

## Data Availability

The data used to support the findings of this study are available from the corresponding author upon request.
